The article "Interferon-gamma deficiency protects against aging-related goblet cell loss" was published in 2016. Journal: Oncotarget.

# Interferon-gamma deficiency protects against aging-related goblet cell loss

**DOI:** 10.18632/oncotarget.11872

**Published:** 2016-09-06

**Authors:** Eugene A. Volpe, Johanna Tukler Henriksson, Changjun Wang, Flavia L. Barbosa, Mahira Zaheer, Xiaobo Zhang, Stephen C. Pflugfelder, Cintia S. de Paiva

**Affiliations:** ^1^ Ocular Surface Center, Department of Ophthalmology, Cullen Eye Institute, Baylor College of Medicine, Houston, Texas, USA; ^2^ Eye Center, Second Affiliated Hospital of Zhejiang University, School of Medicine Zhejiang Provincial Key Laboratory of Ophthalmology, Hangzhou, Zhejiang, China; ^3^ Eye Institute of Xiamen University, Xiamen, Fujian, China

**Keywords:** aging, dry eye, interferon-gamma, goblet cells, IL-17, Gerotarget

## Abstract

Aging is a well-recognized risk factor for dry eye. Interferon-gamma (IFN-γ) has been implicated in conjunctival keratinization and goblet cell loss in dry eye. We investigated the role of IFN-γ in age-related dry eye by evaluating young (8 weeks) and aged (15 months; 15M) C57BL/6 (B6) and IFN-γKO mice. Age effects on the conjunctiva and cornea epithelium were assessed with PAS staining and corneal staining, respectively. Expression of T cell-related cytokines (IL-17A, IFN-γ), chemokines (CXCL10 and CCL20), in the ocular surface epithelium was evaluated by real time PCR. A significant decrease in filled goblet cells was noted in 15M B6 mice and this was significantly lower than age and sex-matched IFN-γKO mice. Aged male B6 had significantly higher IFN-γ, and CXCL10 mRNA in their conjunctiva than female B6 mice. Aged IFN-γKO females had significantly higher IL-17A mRNA in conjunctiva than IFN-γKO males and B6 mice. Corneal barrier dysfunction was observed in 15M female B6 and aged IFN-γKO mice of both sexes; however it was significantly higher in IFN-γKO compared to B6 mice. While there was a significant increase in IL 17A, and CCL20 in corneas of aged female B6 and IFN-γKO mice compared to males, these changes were more evident in aged female IFN-γKO group.

Partial resistance of IFN-γKO mice to aging-induced goblet cell loss indicates IFN-γ is involved in the age-related decline in conjunctival goblet cells. Increased corneal IL-17A expression paralleled corneal barrier disruption in aging female of both strains. IFN-γ appears to suppress IL-17A on the ocular surface.

## INTRODUCTION

Aging is a well-known-risk factor for dry eye. Prevalence of dry eye disease increases with age after the 4^th^ decade and it's more prevalent in women [1-3]. A frequent finding in dry eye is keratinization of the ocular surface epithelium and loss of goblet cells [4-8]. Both IFN-γ and IL-17 have been implicated in the pathogenesis of dry eye associated ocular surface epithelial disease [9-12].

The article "Interferon-gamma deficiency protects against aging-related goblet cell loss" was published in 2016. Journal: Oncotarget.

Alterations in cellular immunity are a known aspect of aging [13]. With increasing age, the thymus begins to shrink, leading to a decrease in the number of naïve T-lymphocytes in the circulation. A compensatory auto proliferation of existing, mature T-cells may lead to the expansion of CD4 positive (^+^) T-cells. These cells are resistant to apoptosis and have been shown to be associated with a variety of autoimmune disorders such as rheumatoid arthritis, multiple sclerosis, and diabetes mellitus [14].

Interferon-gamma (IFN-γ), produced by natural killer, natural killer T cells and T cells, is the signature cytokine of T helper (Th) 1 immune responses and it has been involved in the pathogenesis of colitis and Sjögren Syndrome [15-18]. IFN-γ production by T cells in peripheral blood and conjunctiva progressively increases with age in human studies [19, 20]. There is mounting evidence about a pathogenic role for IFN-γ in dry eye. We have previously shown that desiccating stress decreases goblet cell density mainly to increased IFN-γ, as IFN-γKO mice were resistant to desiccation-induced changes [21]. Subconjunctival injections of IFN-γ or anti-IFN-γ antibody decreased or improved goblet cell density in an experimental dry eye model, respectively [21-24]. IFN-γ produced by NK cells is responsible for upregulation of Th1 cell recruiting chemokines by conjunctival and corneal epithelial cell in experimental dry eye [25, 26]. Cultured conjunctival goblet cells are exquisitely sensitive to IFN-γ, as even minute concentrations of this cytokine promotes goblet cell apoptosis [27]. Increased IFN-γ has been observed in tears and conjunctiva of dry eye patients [9, 12, 28].

IL-17A is the signature cytokine of Th-17 immune responses. It has been implicated in the pathogenesis of several autoimmune diseases, including rheumatoid arthritis, psoriasis and uveitis and inflammatory bowel disease [29-34]. We and others have shown that IL-17A disrupts apical corneal barrier apical function in experimental dry eye [9, 11], by stimulating matrix metalloproteinases that have been implicated in breakdown of epithelial tight junctions [9]. Our published study showed that 24 month-old C57BL/6 mice spontaneously develop a SS-like keratoconjunctivitis sicca, with increased IL-17A and IFN-γ transcript levels in conjunctiva, which was accompanied by loss of conjunctival goblet cells and increased corneal barrier disruption [10]. The role of immune dysfunction in the pathogenesis of age-associated dry eye disease has not been sufficiently investigated.

The purpose of this study was to investigate the roles of IFN-γ and IL-17 in aging and sex-related goblet cell loss and corneal barrier function, respectively. Our studies showed that goblet cell loss in aged IFN-γKO mice was significantly lower than age-matched B6 mice. This was accompanied by increased IFN-γ and IFN-γ inducible-chemokines in the conjunctiva. Increased corneal barrier dysfunction was observed in female mice.

The article "Interferon-gamma deficiency protects against aging-related goblet cell loss" was published in 2016. Journal: Oncotarget.

## RESULTS

### IFN-gamma deficiency reduces aging-related goblet cell loss

One of the hallmarks of aqueous deficient dry eye disease is a decrease in the number of mucin-filled goblet cells [12, 35, 36]. We measured the number of filled goblet cells in 8-week (8W) and 15-month (15M) old B6 and IFN-γKO mice in PAS stained conjunctival sections. There was a significant decrease in the number of PAS^+^ goblet cells in aged B6 mice, compared to 8-week old mice, irrespective of sex (*P* < 0.01, Figure 1A-1B). A significant decrease in GC count was also found in male 15M IFN-KO mice *P* < 0.05, Figure 1A-1B) compared to its baseline, although this was significantly less than the age-related goblet cell loss observed in in B6 mice (∼24% *vs*. 40%, respectively).

**Figure 1:** Aging leads to decreased goblet cell density in C57BL/6 mice **A.** Representative digital images of PAS stained goblet cells (GC) in conjunctiva (purple-magenta cells) of male C57BL/6 and IFN-γ KO mice. Black squares are higher magnification showing goblet cells in details. **B.** Number of PAS^+^ conjunctival GC in C57BL/6 and IFN-γ KO mice of both sexes counted in paraffin-embedded sections. (Mean±SEM, *n* = 5 right eyes). W = weeks; M = male; F = female.

### Age-related increase in T helper (Th) 1 and Th17 associated cytokines in conjunctiva

We have previously shown that T-cell related cytokines are elevated in the conjunctiva of 24 month-old B6 mice [10]. In this study, we evaluated expression of Th1 (*IFN-γ, CXCL10*), Th17 (*IL-17A, CCL20*), and Th2 (*IL-13*) related factors in conjunctiva of young and old mice by real time PCR.

We found that levels of *IFN-γ* mRNA transcript were significantly higher in female B6 mice at 8W (*P* < 0.001) and in male B6 at 15M (*P* < 0.001, Figure 2A), but they were completely absent in the IFN-γKO mice. The mRNA transcripts of *CXCL10*, a chemokine involved in trafficking of Th-1 cells [37], were significantly elevated in the young female B6 mice and aged male B6 mice (*P* < 0.0001, Figure 2B) and were higher in B6 than IFN-γKO in young female and aged male.

CCL20 is a chemokine involved in trafficking of Th-17 cells [38, 39]. *CCL20* and *IL-17A* mRNA transcript levels in conjunctiva were elevated in both young and aged female B6 compared to males (*P* < 0.001). Compared to B6, *CCL20* and *IL-17A* levels were dramatically increased in IFN-γKO mice of both sexes of both ages (*P* < 0.0001, Figure 2C-2D).

The article "Interferon-gamma deficiency protects against aging-related goblet cell loss" was published in 2016. Journal: Oncotarget.

IL-13 is a cytokine that promotes goblet cell homeostasis [40, 41]. IL-13 mRNA transcript levels were higher in female 8W B6 and male 15M B6 (*P* < 0.0001, Figure 2E), and at the same time were significantly higher in IFN-γKO female mice, in both young and aged groups (*P* < 0.0001). IL-13/IFN-γ mRNA ratio was decreased in aged male B6, while IFN-γKO mice had unchecked IL-17 and IL-13 (Figure 2F and not shown).

**Figure 2:** Aging induces sex and age specific findings in conjunctiva Relative fold of mRNA expression of IFN-γ **A.** and CXCL10 **B.**, IL-17A **C.**, CCL20 **D.**, IL-13 **E.**, and IL-13/IFN-γ ratio in conjunctiva in B6 mice **F.** Bar graphs show mean ± SEM (*n* = 6 animals, conjunctiva from both eyes of the same animal were pooled into one sample, yielding a final sample size of 6). W = weeks; M = male; F = female; * *P* < 0.05; ** *P* < 0.01; *** *P* < 0.001; **** *P* < 0.0001; sex comparison at same age.

### Decreased corneal barrier function in aged female mice

Increased corneal permeability to fluorescent dyes is another hallmark of dry eye. Antibody neutralization of IFN-γ itself or of IFN-γ-producing NK cells has been shown to protect against developing corneal staining in a murine dry eye model [24, 26]. We compared corneal permeability to the 70kDa fluorescent molecule Oregon-Green Dextran (OGD) of young and aged B6 and IFN-γKO mice of both sexes. Sex-specific differences were observed; aged female B6 had increased corneal barrier disruption which was not observed in age-matched male B6 mice (Figure 3A-3B). IFN-γKO mice of both sexes had increased uptake of OGD dye with aging; however, similar to B6 mice, these changes were more pronounced in females. Moreover, corneal permeability in 15M female IFN-γKO mice was also significantly increased compared to 15M B6 mice.

**Figure 3:** Corneal barrier function in C57BL/6 and IFN-γKO mice of both sexes at 8 weeks and 15 months of age **A.** Representative digital images of Oregon Green dextran (OGD) corneal staining that were used to generate the bar graphs in B. **B.** Corneal Oregon Green dextran (OGD) fluorescence intensity score (mean±SEM, *n* = 15 animals). W = weeks; M = male; F = female; * *P* < 0.05; ** *P* < 0.01; *** *P* < 0.001; **** *P* < 0.0001; sex comparison at same age.

### Age-related increase in T-cell associated cytokines in cornea

IL-17A and matrix-metalloproteinase −9 (MMP-9) have been found to participate in desiccation-induced corneal barrier disruption [9, 11, 42]. We hypothesized that aged-related corneal barrier disruption would be accompanied by an increase in the same factors as those previously observed in inducible dry eye models. Therefore, we compared the expression of *IL-17A, CCL20* and *MMP-9*, in corneas of aged mice to young mice of both groups by real-time PCR.

The article "Interferon-gamma deficiency protects against aging-related goblet cell loss" was published in 2016. Journal: Oncotarget.

In B6 mice, *IL-17A* mRNA transcript levels were elevated only in aged females (*P* < 0.001), and they were dramatically increased in IFN-γKO mice of both sexes (*P* < 0.001) and particularly in young and old (*P* < 0.0001, Figure 4A). *CCL20* mRNA transcript level in cornea was elevated in the both young and aged female B6 mice (*P* < 0.0001), and significantly increased in young IFN-γKO mice of both sexes (*P* < 0.0001) and in aged IFN-γKO female mice (*P* < 0.0001; Figure 4B). MMP-9 has been shown to mediate corneal barrier disruption in dry eye [42]. *MMP-9* mRNA transcript levels were significantly elevated in aged female B6 cornea compared to young mice (*P* < 0.0001), and significantly higher in female IFN-γKO mice, in both young (*P* < 0.0001) and aged (*P* < 0.05) groups (Figure 4C).

**Figure 4:** Aging increases IL-17, CCL20 and MMP-9 mRNA expression in cornea Relative fold of mRNA expression of IL-17A **A.**, CCL20 **B.** and MMP-9 **C.** in corneal epithelium. Bar graphs show mean ± SEM (*n* = 6, corneal epithelium pooled from both eyes of the same animal). W = weeks; M = male; F = female; * *P* < 0.05; ** *P* < 0.01; *** *P* < 0.001; **** *P* < 0.0001; sex comparison at same age.

## DISCUSSION

Dry eye is a very prevalent disease in the aging population [1, 2]. It is estimated that dry eye is one of the top reasons for seeking eye care, mostly because corneal barrier disruption is responsible for irritation and decreased vision [43, 44]. Among dry eye patients, 11% have been estimated to have the systemic autoimmune condition Sjögren Syndrome [45, 46], a severe and potentially blinding condition. Strong correlation between age and female sex and prevalence of DED has been well established [2, 47]. However, the exact mechanisms why dry eye is more prevalent in aged women have not been elucidated yet.

Goblet cells are highly secretory epithelial cells that are abundant in conjunctiva, and digestive tract. Cornification and goblet cell loss in the conjunctival epithelium has been recognized in dry eye patients for over than three decades [8, 12, 48, 49]. Our previous studies showed that 24-month old B6 mice of both sexes had a decreased number of mucin-filled goblet cells [10]. This was accompanied by increased IFN-γ expression, leading us to hypothesize that IFN-γ may contribute to the goblet cell loss in aged mice. Our current study demonstrated that IFN-γKO mice had a significantly less goblet cells loss than age-matched B6 mice. The decline in goblet cells was accompanied by increased IFN-γ and CXL10 expression in the conjunctiva of B6 mice. Interestingly, aged female B6 and IFN-γKO mice displayed greater corneal barrier disruption and increased IL-17A and CCL20 mRNA levels in cornea than aged male mice.

The article "Interferon-gamma deficiency protects against aging-related goblet cell loss" was published in 2016. Journal: Oncotarget.

Our findings indicated that IFN-γ is partially responsible for aging-related goblet cell loss. Williams and colleagues showed an age-related increase in IFN-γ-producing CD4^+^ T cells in conjunctiva of human subjects [20]. Recent studies have shown a close relationship between the mucosal immune system and conjunctival goblet cells, a relationship that has been identified in other mucosal tissues, including the intestine and airways [50, 51]. Studies in the lung have demonstrated that IL-13 induces goblet cell hyperplasia [52, 53]. In the conjunctiva, goblet cell differentiation and MUC5AC production is reciprocally regulated by the T helper cytokines IFN-γ and IL-13 [21, 27, 40, 41]. We have shown that IL-13 has a homeostatic role in maintaining conjunctival goblet cells, whereas IFN-γ promotes conjunctival cornification and goblet cell loss [21, 24]. IL-13KO mice have decreased goblet cell density at baseline and subconjunctival injections of IL-13 during experimental dry eye rescued goblet cell density compared to placebo-injected mice [40]. We have also shown that IL-13 -stimulated cultured conjunctival goblet cells have increased proliferation and production of Muc5ac and Muc2 [41]. Prior studies from our laboratory showed that IFN-γKO mice were resistant to desiccation-induced goblet cell loss and subconjunctival administration of IFN-γ in IFN-γKO mice decreased goblet cell to similar levels as wild-type mice [21], as well as upregulated cornified envelope proteins that also increase in dry eye [4]. We have also demonstrated that subconjunctival injections of anti-IFN-γ during desiccating stress prevented goblet cell loss [24]. We also discovered that IFN-γ causes endoplasmic reticulum stress and induces an unfolded protein response in cultured conjunctival goblet cells, as a molecular mechanism responsible for the reduced mucin secretion induced by IFN-γ [27]. Our primary conjunctival cultures are exquisitely sensitive to IFN-γ as even minute concentrations of this cytokine decreased proliferation, inhibited synthesis of mature mucins and induced profound morphological changes, despite increased levels of mucin gene transcripts [27]. Taken together, these results indicate a critical role for IFN- in conjunctival goblet cell loss/dysfunction, *in vitro*, and in two different models of dry eye, including aging and desiccating stress in young mice.

The article "Interferon-gamma deficiency protects against aging-related goblet cell loss" was published in 2016. Journal: Oncotarget.

IL-17A has also been noted to increase in mice and humans with aging and to participate in autoimmunity [54-57]. IL-17A has been shown to cause epithelial barrier disruption in mice [9, 11] and to increase expression of MMPs [58, 59]. MMP-induced lysis of tight junctions and desquamation of the corneal epithelium is responsible for corneal barrier disruption in dry eye [42]. The discovery of Th-17 cells has challenged the Th1/Th2 paradigm of cross regulation of autoimmunity. While IFN-γ has been shown to inhibit the development of IL-17-producing effector CD4^+^ T cells *in vitro* [60, 61], an *in vivo* suppressive effect of IFN-γ on IL-17 production has not been clearly demonstrated. Both Th1 and Th17 cells are pathologic in some experimental models, such as experimental autoimmune uveitis, dry eye and rheumatoid arthritis [62-67]. In the collagen-induced arthritis model, young IFN-γKO B6 mice produced higher levels of IL-17 in response to immunization with type II collagen compared to wild-type B6 mice [68]. Anti-IL-17 antibody prevented collagen-induced arthritis in the IFN-γ-receptor KO, which has elevated levels of IL-17 compared to wild-type mice [64]. Antibody depletion of IL-17 prior to and during desiccating stress did not increase IFN-γ mRNA in conjunctiva [9]. Here we report that suppression of IL-17A by IFN-γ occurs naturally even in young mice, but a significant clinical phenotype (corneal barrier disruption) is only found with advanced aging, demonstrating that a certain accumulation of still unknown events is necessary for a full dry eye phenotype. Interestingly, greater age-related corneal barrier disruption was observed in female mice. This is in agreement with a recent study demonstrating that young female B6 mice are more susceptible to corneal barrier disruption in a desiccating environment and have greater levels of IL-17 in draining lymph nodes and lacrimal gland than young male mice subjected to the same protocol [69]. IL-17 mRNA levels in corneal epithelia peaked at the same time as maximum corneal barrier disruption in the 8-week old CD25 (IL-2 receptor alpha) knock-out mouse model of Sjögren Syndrome [33]. Our group was the first to describe that aged female B6 mice spontaneously develop corneal barrier disruption [10]. Increased levels of IL-17A have been reported in both tears and conjunctiva of dry eye patients. [9, 70-72]. In humans, dry eye disease affects both sexes, but it has a great incidence in female patients [1, 2, 73-75]. We can speculate that increased corneal disease and increased IL-17 in females may be one of the reasons why dry eye is more prevalent in female sex, but further studies are necessary to investigate this correlation.

The article "Interferon-gamma deficiency protects against aging-related goblet cell loss" was published in 2016. Journal: Oncotarget.

In conclusion, this study provides evidence that IFN-γ actively participates in aging-related conjunctival goblet cell loss and also provides insights about the complex cytokine interactions in dry eye pathogenesis. Therapies targeting both IFN-γ and IL-17A cytokines may be needed to fully address the spectrum of dry eye manifestations and to improve the quality of visual function and life of an aging population.

## MATERIALS AND METHODS

### Animals

This research protocol was approved by the Baylor College of Medicine Center for Comparative Medicine, and it conformed to the standards of the Association for Research in Vision and Ophthalmology Statement for the Use of Animals in Ophthalmic and Vision Research. C57BL/6 (B6), IFN-γKO (B6.129S7-ifng^tm1Ts^/J, on a B6 background) mice of both sexes were purchased from Jackson Laboratories (Bar Harbor, ME) for establishing breeding colonies in our facility and were used at 8 weeks and 15 months of age. Offspring mice housed in our vivarium until they reach appropriate age. Twenty-six mice per age/strain/sex were used: five for histologic sections, 15 for measuring corneal permeability, six for gene analysis.

### Corneal permeability to oregon-green dextran

Corneal epithelial permeability to Oregon-Green dextran [OGD; 70 000 molecular weight (MW); Invitrogen, Eugene, OR, USA] was assessed at 8 weeks and 15 months in both sexes and strains (C57BL/6 and IFN-γKO) as previously described [9]. Briefly, 0.5 ml of 50μg/ml OGD was instilled onto the ocular surface 1 min before euthanasia. Corneas were rinsed with 2 μl of phosphate buffered saline (PBS) and photographed with a stereoscopic zoom microscope (model SMZ 1500; Nikon, Melville, NY, USA), under fluorescence excitation at 470 nm. The severity of corneal OGD staining was digitally graded as previously reported [9]. The mean fluorescence intensity measured inside the 2-mm central zone by the image analysis software (NIS Elements, version 3.0, Nikon, Melville, NY) was transferred to a database and the results averaged within each group.

### Histology, periodic acid schiff staining

Five right eyes from each sex, at 8W and 15M, were surgically excised, fixed in 10% formalin, paraffin embedded, and 8-μm sections were cut. Ocular sections were cut at the center of the eye, where the lens has its maximum diameter. Sections were stained with H&E for evaluating morphology and with periodic-Schiff (PAS) reagent for measuring goblet cell density. The superior and inferior conjunctiva were examined and photographed with a microscope equipped with a digital camera (Eclipse E400 with a DS-Fi1; Nikon, Melville, NY, USA). The number of goblet cells in the superior and inferior conjunctiva was measured in 3 sections from each eye that were at least 300 μm apart, using image-analysis software (NIS Elements Software, version 3.0, BR, Nikon) and expressed as number of goblet cells per mm as previously reported [21].

The article "Interferon-gamma deficiency protects against aging-related goblet cell loss" was published in 2016. Journal: Oncotarget.

### RNA isolation and real-time PCR

Total RNA from the cornea and conjunctiva was collected as previously described [9] and extracted using a Qiagen RNeasy Plus^®^ Micro RNA isolation Kit (Qiagen, Valencia, CA) according to the manufacturer's instructions, quantified by a NanoDrop^®^ ND-1000 Spectrophotometer (Thermo Scientific, Wilmington, DE) and stored at −80°C. Six samples per group/age were used, and 1 sample consisted of pooled conjunctiva or cornea of right and left eyes of the same animal. The RNA concentration was measured by its absorption at 260 nm and samples were stored at −80°C until use. First-strand cDNA was synthesized with random hexamers by M-MuLV reverse transcription (Ready-To-Go You-Prime First-Strand Beads; GE Healthcare, Inc., Arlington Heights, NJ), as previously described [9]. Real-time PCR was performed with specific MGB probes (Taqman; Applied Biosystems, Inc., Foster City, CA) and PCR master mix (Taqman Gene Expression Master Mix), in a commercial thermocycling system (StepOnePlus Real-Time PCR System, Applied Biosystems), according to the manufacturer's recommendations. Murine MGB probes were *HPRT1* (Mm00446968), *CCL20* (Mm00444228), *CXCL10* (Mm445235), *IFN-γ* (Mm00801778), *IL-13* (Mm99999190), *IL-17A* (Mm00439618) and *MMP-9* (Mm00442991). The *HPRT1* gene was used as an endogenous reference for each reaction. The results of quantitative PCR were analyzed by the comparative C_T_ method where target change = 2^ΔΔCT^. The results were normalized by the C_T_ value of HPRT1. The mean C_T_ of relative mRNA level in the eight week male group was used as the calibrator.

### Statistical analysis

Two-way analysis of variance (ANOVA) or the Kruskall-Wallis tests were used for overall statistical comparisons, followed by Sidak's multiple comparison test. *P* < 0.05 was considered statistically significant. These tests were performed using GraphPad Prism 6.0 software (GraphPad Software, Inc., San Diego, CA).

## Abbreviations

ANOVA: analysis of variance
APC: antigen-presenting cells
CCL20: CC-chemokine attractant ligand 20
CXCL10: C-X-C motif chemokine ligand 10 (or IP-10: IFN-γ inducible protein 10)
DED: dry eye disease
GC: goblet cells
HPRT1: hypoxanthine phosphoribosyltransferase 1 gene
IFN-γ: interferon-gamma
IL: interleukin
MGB: 3′-minor groove binder-DNA probes
MGD: meibomian gland disease
MHC: major histocompatibility complex
MMPs: matrix metallo-proteinases
M-MuLV: Moloney murine leukemia virus
MUC5AC: mucin 5AC gene with protein product
OCT: optimal cutting temperature compound
OGD: Oregon Green dextran
PBS: phosphate-buffered saline;
RT-PCR: real-time polymerase chain reaction.
